The article "SNHG1/miR-145-5p/KLF5 Axis Participates in Regulating the Proliferation and Migration of Oral Squamous Cell Cancer" was retracted in 2023. Reasons: suspected computer-generated content; unreliable results or conclusions; concerns about the data; concerns about the results or conclusions.

# SNHG1/miR-145-5p/KLF5 Axis Participates in Regulating the Proliferation and Migration of Oral Squamous Cell Cancer

**DOI:** 10.1155/2022/2053271

**Published:** 2022-03-03

**Authors:** Haiyan Xin, Ziyan Feng, Chao Yao

**Affiliations:** ^1^Department of Orthodontics, Central Laboratory of Jinan Stamotological Hospital, Jinan Key Laboratory of Oral Tissue Regeneration, Jinan 250001, Shandong, China; ^2^Fuzhou Medical College of Nanchang University, Fuzhou 344000, Jiangxi, China; ^3^Department of Oral and Maxillofacial Surgery, Central Laboratory of Jinan Stamotological Hospital, Jinan Key Laboratory of Oral Tissue Regeneration, Jinan 250001, Shandong, China

## Abstract

We aimed to clarify the molecular mechanism of lncRNA SNHG1 in regulating the OSCC process. Clinical samples of OSCC were collected for detecting the differential level of SNHG1 by qRT-PCR. Pathological indexes of OSCC patients were analyzed for uncovering the prognostic value of SNHG1. The interaction between SNHG1 and miR-145-5p was assessed through the bioinformatics method and dual-luciferase reporter assay. Their coregulation on proliferative and migratory functions of Tca8113 and CAL-27 cells was explored by the CCK-8, EdU, and Transwell assay. Finally, the regulatory effect of miR-145-5p on its downstream gene KLF5 was evaluated. SNHG1 was abnormally upregulated in OSCC samples and linked to a poor prognosis of OSCC patients. Serving as an oncogene, SNHG1 strengthened proliferative and migratory functions of Tca8113 and CAL-27 cells. miR-145-5p was a key downstream target inducing the oncogenic role of SNHG1 in the OSCC process with KLF5 as its downstream gene. SNHG1/miR-145-5p/KLF1 axis is responsible for driving the malignant process of OSCC.

## 1. Introduction

Oral squamous cell carcinoma (OSCC) is the eighth most common cancer in the world, with more than 300,000 new cases each year [1]. Despite the great improvement made on therapeutic strategies, the 5-year survival of OSCC is lower than 50% mainly because of lymphatic metastasis [2]. Both radiotherapy and chemotherapy can be effective for OSCC patients. Nevertheless, the emergence and development of drug resistance largely limit therapeutic efficacy [3]. Abundant evidence has supported the fact that dysfunction of oncogenes and tumor-suppressor genes is of significance in the cancer process.

Long noncoding RNAs (lncRNAs) are 200-nucleotide long, noncoding RNAs with barely or no protein-encoding function [4, 5]. They are widely involved in the cancer process [6, 7]. It is reported that TP73-AS1 is able to protect bladder cancer from the malignant development and predicts its prognosis [8]. EPEL participates in the activation of the E2F signaling in lung cancer [9]. Previously, SNHG1 is determined to enhance proliferative and migratory capacities of cervical cancer cells [10]. As a vital regulator, SNHG1 is capable of regulating miR-151-5p and EZH2, thus mediating colorectal carcinoma process [11]. The role of SNHG1 in the OSCC process is rarely reported. Our study identified an important feedback loop through the bioinformatics method and mainly explored its potential effect on regulating OSCC cell functions.

## 2. Materials and Methods

### 2.1. Subjects and Samples

A total of 31 OSCC patients treated in our hospital were retrospectively analyzed, including 21 men and 10 women. Their paired OSCC tissues and normal ones were collected and stored at −80°C. Tumor staging was determined based on the Union for International Cancer Control (UICC) criteria. Recruited eligible OSCC patients were pathologically confirmed, and they did not receive preoperative anticancer treatment. Subjects with other malignancies were excluded. This study was approved by the research ethics committee of our hospital and complied with the Helsinki Declaration. Informed consent was obtained from subjects and their parents.

### 2.2. Quantitative Real-Time Polymerase Chain Reaction (qRT-PCR)

Tissue samples were processed by TRIzol (Invitrogen, Carlsbad, CA, USA) for isolating RNAs. After purification, qualified RNAs (RNA concentration >210 ng/*μ*L and A260/280 = 1.8–2.1) were reversely transcribed to complementary deoxyribonucleic acids (cDNAs) and subjected to qRT-PCR using SYBR^®^ Premix Ex Taq^™^ (Takara, Tokyo, Japan) at 95°C for 1 min, followed by 40 cycles at 95°C for 10 s, 64°C for 30 s, and 72°C for 30 s. Relative levels of PCR products were calculated by 2^−ΔΔCt^ and normalized to those of glyceraldehyde 3-phosphate dehydrogenase (GAPDH).

### 2.3. Cell Culture

OSCC cell lines (FaDu, SCC-25, CAL-27, and Tca8113) and epithelial cells of oral mucosa (OMECs) were provided by Cell Bank, Shanghai Institute for Biological Sciences (Shanghai, China). Cells were cultured in Dulbecco's Modified Eagle Medium (DMEM) (Gibco, Rockville, MD, USA) containing 10% fetal bovine serum (FBS) (Gibco, Rockville, MD, USA) at 37°C and 5% CO_2_. Cell passage was conducted at a ratio of 1 : 3, with an interval of 2 days.

### 2.4. Transfection

Transfection plasmids were synthesized by GenePharma (Shanghai, China). Cells were cultured to 50–60% confluence in a 6-well plate and transfected using Lipofectamine 2000 (Invitrogen, Carlsbad, CA, USA). After 48 h transfection, cells were collected for verifying transfection efficacy and functional experiments.

### 2.5. 5-Ethynyl-2'-deoxyuridine (EdU) Assay

Cells were induced with 50 *μ*M EdU (RiboBio, Guangzhou, China) for 2 h and dyed using AdoLo and 4',6-diamidino-2-phenylindole (DAPI) in the dark. EdU-labeled cells were captured for calculating the percentage of EdU incorporation.

### 2.6. Dual-Luciferase Reporter Assay

XhoI and NotI digestion sites were added on both ends of target gene sequences of SNHG1-WT and SNHG1-MUT, and they were cloned into PUC-T vectors. After enzyme digestion for 2 h, sequences were electrophoresed. Purified products, alongside psiCHECK-2 vectors, were induced with DH5*α* receptive cells that were cultivated in an ice bath. They were then subjected to heat shock in a water bath at 42°C for 60 s. The mixture was quickly placed on ice for 3 min, followed by incubation with 500 *μ*L of LB and shaking at 37°C, 200 r/min for 1 h. The obtained bacteria fluid was applied on the LB solid medium containing ampicillin and cultivated overnight. On the other day, colonies were electrophoresed, purified, and analyzed. The target colonies were subjected to amplification culture for isolating plasmid DNA. They were cotransfected in cells with the miR-145-5p inhibitor or negative control for 24 h, followed by the measurement of luciferase activity (Promega, Madison, WI, USA).

### 2.7. Cell Counting Kit-8 (CCK-8) Assay

Cells were inoculated in a 96-well plate with 2 × 10^3^ cells/well. At 0, 24, 48, and 72 h, optical density at 450 nm of each sample was recorded using the CCK-8 kit (Dojindo Laboratories, Kumamoto, Japan) for plotting the viability curves.

### 2.8. Transwell Migration Assay

200 *μ*L of suspension (2 × 10^5^ cells/mL) was applied on the top of a Boyden chamber precoated with 200 *μ*L of diluted Matrigel (Corning, Corning, NY, USA), which was placed in each well containing 700 *μ*L of the medium and 20% FBS. Cells were allowed to migrate for 48 h, and they were fixed, dyed, and captured for counting in five random fields per sample.

### 2.9. Statistical Analysis

GraphPad Prism 7 (La Jolla, CA, USA) was used for statistical analyses, and data were expressed as mean ± standard deviation. Differences between groups were compared by the *t*-test. Survival analysis was conducted by the Kaplan–Meier method. Correlation between expression levels of two genes was assessed by Pearson's correlation test. *P* < 0.05 was considered as statistically significant.

## 3. Results

### 3.1. Upregulation of SNHG1 in OSCC

A total of 31 pairs of OSCC and normal tissues were collected for detecting differential levels of SNHG1. Compared with controls, SNHG1 was significantly upregulated in OSCC tissues (Figure 1(a)). Classified by metastasis status, a higher level of SNHG1 was detected in metastatic OSCC cases in comparison to nonmetastatic ones (Figure 1(b)). Survival analysis uncovered that OSCC patients expressing a high level of SNHG1 suffered worse survival in comparison to patients expressing a low level of SNHG1 (Figure 1(c)). In OSCC cell lines, SNHG1 was consistently upregulated (Figure 1(d)). It is suggested that SNHG1 was upregulated in OSCC samples and predicted a poor prognosis.

### 3.2. Knockdown of SNHG1 Decreased Proliferative and Migratory Abilities of OSCC

Transfection of si-SNHG1 significantly downregulated SNHG1 in Tca8113 and CAL-27 cells, yielding a transfection efficacy of over 70% (Figure 2(a)). Proliferative ability of OSCC cells was assessed by the CCK-8 and EdU assay. Knockdown of SNHG1 in Tca8113 and CAL-27 cells not only reduced cell viability but also EdU-positive rate, indicating the weakened proliferative function (Figures 2(b)–2(d)). In addition, results of the Transwell assay showed that knockdown of SNHG1 attenuated migratory function in OSCC cells (Figure 2(e)). Collectively, SNHG1 was able to stimulate proliferative and migratory potentials of OSCC cells.

### 3.3. miR-145-5p Was the Target Gene of SNHG1

Through searching lncRNASNP2, a binding site in the miR-145-5p 3'UTR was emerged that paired to the SNHG1 3'UTR (Figure 3(a)). Luciferase vectors were synthesized based on the predicted binding site. Knockdown of miR-145-5p remarkably upregulated SNHG1 in CAL-27 and Tca8113 cells (Figure 3(b)). Later, data from the dual-luciferase reporter assay confirmed the binding between SNHG1 and miR-145-5p (Figures 3(a) and 3(d)). Compared with normal ones, miR-145-5p was downregulated in OSCC tissues, displaying a negative correlation to that of SNHG1 (Figures 3(e) and 3(f)).

### 3.4. miR-145-5p Induced the Oncogenic Role of SNHG1 in OSCC

To further analyze the involvement of miR-145-5p in the OSCC process, miR-145-5p knockdown was achieved by transfection of the miR-145-5p inhibitor (Figure 4(a)). In comparison to OSCC cells with SNHG1 knockdown only, viability and EdU-positive rate were both lower in those with coknockdown of SNHG1 and miR-145-5p (Figures 4(b)–4(d)). Moreover, a higher migratory cell number in OSCC cells was detected in those with coknockdown of SNHG1 and miR-145-5p than the si-SNHG1 group (Figure 4(e)). It is indicated that miR-145-5p was responsible for the oncogenic role of SNHG1 in OSCC.

### 3.5. miR-145-5p Could Bind the Oncogenic Gene KLF5

Binding sequences in the 3'UTR of miR-145-5p and KLF5 were predicted using TargetScan (Figure 5(a)). Their binding relationship was further verified by the dual-luciferase reporter assay (Figures 5(b) and 5(c)). In comparison to normal tissues, KLF5 was highly expressed in OSCC tissues (Figure 5(d)). Its level was upregulated in CAL-27 and Tca8113 cells transfected with the miR-145-5p inhibitor (Figure 5(e)). Taken together, miR-145-5p could negatively regulate the oncogenic gene KLF5 and induce the oncogenic role of SNHG1 in the OSCC process.

## 4. Discussion

A growing number of evidence has demonstrated the important functions of lncRNAs in pathological processes [12]. Our study detected an abnormal upregulation of SNHG1 in clinical samples of OSCC. By analyzing clinical data of recruited patients, a higher level of SNHG1 was detected in metastatic OSCC cases in comparison to nonmetastatic ones. Moreover, Kaplan–Meier curves obtained the conclusion that SNHG1 was an unfavorable factor to the survival of OSCC. Subsequently, *in vitro* experiments uncovered that SNHG1 was able to enhance proliferative and migratory functions of OSCC cells. We believed that SNHG1 exerted an oncogenic role in the OSCC process. Its specific molecular mechanism, however, was unclear.

Using online bioinformatics software, we predicted a binding site in the miR-145-5p 3'UTR pairing to that of SNHG1. Later, dual-luciferase reporter assay confirmed their binding. In a previous study, SNHG1 is identified to stimulate the invasiveness of breast cancer by sponging miR-382 [1]. It activates the Wnt signaling in NSCLC through exerting the miRNA sponge effect on miR-101-3p [13]. Our study, for the first time, discovered a potential interaction between SNHG1 and miR-145-5p, and we verified their coregulation on triggering the OSCC process. In multiple types of cancers, miR-145-5p serves as an anticancer gene [14–16]. In addition, miR-145-5p has a close relation to cell apoptosis, and it can be utilized as a therapeutic target for oral cancer [17]. miR-145-5p has several target genes. Among them, KLF5 is considered as the key factor for inducing differentiation of oral cancer cells [18]. KLF5 is also an intracellular transcription factor involved in signal transduction [19]. Dysregulation of KLF5 can lead to abnormal changes in Wnt, Ras, TGF*β*, Hippo, Notch signaling, sulfonic acid receptors, or hormone receptors in tumors, eventually leading to carcinogenesis [20]. Its diverse biological functions endow the potential as a famous target for cancer treatment [21]. In the present study, KLF5 was verified to be the downstream gene binding miR-145-5p. Taken together, we have discovered a feedback loop SNHG5/miR-145-5p/KLF5 that is responsible for aggravating the OSCC process through strengthening malignant proliferative and migratory functions. Our findings provide a novel option for developing targeted therapy of OSCC.

## 5. Conclusions

SNHG1/miR-145-5p/KLF1 axis is responsible for driving the malignant process of OSCC.

## Figures and Tables

**Figure 1:** Upregulation of SNHG1 in OSCC. (a) Upregulated SNHG1 in OSCC tissues. (b) SNHG1 was highly expressed in metastatic OSCC cases. (c) SNHG1 predicted a poor prognosis of OSCC. (d) Upregulated SNHG1 in OSCC cell lines. ^*∗*^*P* < 0.05, ^*∗∗*^*P* < 0.01, and ^*∗∗∗*^*P* < 0.001.

**Figure 2:** Knockdown of SNHG1 decreased proliferative and migratory abilities of OSCC. (a) Transfection efficacy of si-SNHG1 in Tca8113 and CAL-27 cells. (b, c) Transfection of si-SNHG1 reduced viability in Tca8113 and CAL-27 cells. (d) Transfection of si-SNHG1 reduced EdU-positive rate in Tca8113 and CAL-27 cells. (e) Transfection of si-SNHG1 reduced migration in Tca8113 and CAL-27 cells (200x). ^*∗*^*P* < 0.05 and ^*∗∗*^*P* < 0.01.

**Figure 3:** miR-145-5p was the target gene of SNHG1. (a) Binding site in the 3'UTR of miR-145-5p and SNHG1. (b) SNHG1 level was upregulated in Tca8113 and CAL-27 cells transfected with the miR-145-5p inhibitor. (c, d) Luciferase activity in Tca8113 and CAL-27 cells coregulated by miR-145-5p and SNHG1. (e) Downregulated miR-145-5p in OSCC tissues. (f) A negative correlation between miR-145-5p and SNHG1 levels in OSCC tissues. ^*∗∗*^*P* < 0.01 and ^*∗∗∗*^*P* < 0.001.

**Figure 4:** miR-145-5p induced the oncogenic role of SNHG1 in OSCC. (a) Transfection efficacy of the miR-145-5p inhibitor in Tca8113 and CAL-27 cells. (b, c) Cotransfection of si-SNHG1 and miR-145-5p inhibitor reversed the reduced viability in Tca8113 and CAL-27 cells with SNHG1 knockdown. (d) Cotransfection of si-SNHG1 and miR-145-5p inhibitor reversed the reduced EdU-positive rate in Tca8113 and CAL-27 cells with SNHG1 knockdown. (e) Cotransfection of si-SNHG1 and miR-145-5p inhibitor reversed the reduced migration in Tca8113 and CAL-27 cells with SNHG1 knockdown (200x). ^*∗*^*P* < 0.05 and ^*∗∗*^*P* < 0.01 vs. the si-NC group; ^#^*P* < 0.05 and ^##^*P* < 0.01 vs. the si-SNHG1 group.

**Figure 5:** miR-145-5p could bind the oncogenic gene KLF5. (a) Binding site in the 3'UTR of miR-145-5p and KLF5. (b, c) Luciferase activity in Tca8113 and CAL-27 cells coregulated by miR-145-5p and KLF5. (d) Upregulated KLF5 in OSCC tissues. (e) KLF5 was upregulated in Tca8113 and CAL-27 cells transfected with the miR-145-5p inhibitor. ^*∗∗*^*P* < 0.01.

## Data Availability

The datasets used and analyzed during the current study are available from the corresponding author upon reasonable request.
